The article "Antimicrobial Effects of Gum Arabic-Silver Nanoparticles against Oral Pathogens" was published in 2022. Journal: Bioinorg Chem Appl.

# Antimicrobial Effects of Gum Arabic-Silver Nanoparticles against Oral Pathogens

**DOI:** 10.1155/2022/9602325

**Published:** 2022-12-13

**Authors:** Omnia Ahmed, Nicole R. S. Sibuyi, Adewale O. Fadaka, Abram M. Madiehe, Ernest Maboza, Annette Olivier, Mervin Meyer, Greta Geerts

**Affiliations:** ^1^Department of Restorative Dentistry, Faculty of Dentistry, University of the Western Cape, Bellville, South Africa; ^2^Department of Science and Innovation (DSI) ‐ Mintek Nanotechnology Innovation Centre (NIC) Biolabels Research Node, Department of Biotechnology, University of the Western Cape, Bellville, South Africa; ^3^Oral and Dental Research Laboratory, Faculty of Dentistry, University of the Western Cape, Bellville, South Africa

## Abstract

Dental caries is considered one of the most prevalent oral diseases worldwide, with a high rate of morbidity among populations. It is a chronic infectious disease with a multifactorial etiology that leads to the destruction of the dental tissues. Due to their antimicrobial, anti-inflammatory, antifungal, and antioxidant properties; silver nanoparticles (AgNPs) are incorporated in dental products to help prevent infectious oral diseases. In this study, the antimicrobial effects of AgNPs synthesized using Gum Arabic extracts (GAE) were examined. The GA-AgNPs were synthesized and characterized using ultraviolet-visible (UV-Vis) spectrophotometer, dynamic light scattering (DLS), transmission electron microscopy (TEM), and Fourier transform infrared (FTIR) spectroscopy. The antimicrobial activity of the GA-AgNPs was evaluated on *Streptococcus sanguinis* (*S*. *sanguinis*), *Streptococcus mutans* (*S*. *mutans*), *Lactobacillus acidophilus* (*L*. *acidophilus*), and *Candida albicans* (*C*. *albicans*) using agar disc diffusion and microdilution assays. The antibiofilm of GA-AgNPs was evaluated on the surface of human tooth enamel that had been exposed to *S*. *mutans* with and without the GA-AgNPs using scanning electron microscopy (SEM). GA-AgNPs were spherical in shape with a particle size distribution between 4 and 26 nm. The GA-AgNPs exhibited antimicrobial activity against all the tested oral microbes, with GA-AgNPs_0.4g having higher antimicrobial activity. The GA-AgNPs_0.4g inhibited *S*. *mutans* adhesion and biofilm formation on the surface of the tooth enamel. Therefore, this study supports the prospective implementation of the plant extract-mediated AgNPs in dental healthcare.

## 1. Introduction

Phytotherapy, i.e. the use of herbs or plant extracts to manage health, has played an important role in medicine for centuries. In fact, a significant number of drugs in clinical use are of plant origin or are inspired by plant-based products [1, 2]. Examples include cancer chemotherapeutic drugs such as paclitaxel, a dipertene isolated from the *Taxus brevifolia* Nutt bark extracts [2]; and camptothecin from the *Camptotheca acuminate* stem [3]. Similarly, products for oral health and hygiene were developed from the use of plant products [4–6], where chewing sticks resulted in toothbrushes [5], plant-based decoctions into mouthwash, varnish, and remineralization agents. These traditional practices are still used in lower income areas to date. In addition, some of the herbal remedies such as propolis, and clove are incorporated into commercial oral health-promoting products such as toothpaste, varnish, and irrigants [4, 7]. Over the years, several plant species with oral health promoting properties have been identified. These include plant products made from medicinal plants (aloe vera), vegetables (garlic), herbs/spices (turmeric), fruits (pomegranate), and so on. [8]. Their application in dentistry is encouraged for their varied biological benefits, particularly, their anti-inflammatory, analgesic, antimicrobial, antiplaque, antigingivitis, and antioxidant properties, all of which are attributed to the various phytochemicals present in those plant extracts [4, 5, 7–10].

There has been renewed interest in plant extracts as a source of bioactive agents [11] for the treatment of diseases, including oral infections. Plant products have demonstrated low side effects compared to commercial chemical agents [12]. In search of novel antimicrobial agents against certain pathogenic species causing plaque formation and tooth decay, GA has shown promising results [13]. GA is an exudate acquired from the stem and branches of Acacia tree species [14]. It contains minerals such as calcium, magnesium, and potassium [15]. Therefore, GA is considered a prebiotic agent, promoting the growth or activity of microbes that support the health of the host [16]. GA has been proven to alleviate digestive discomfort, reduce inflammation in the intestinal mucosa [17], and has been implicated in the treatment of both chronic renal failure and diabetes [18, 19]. As an oral hygiene agent, GA may enhance remineralization of caries due to its high concentration of calcium [13] and inhibits early deposition of dental plaque [20]. Moreover, GA inhibits growth of certain pathogenic periodontal species such as *Porphyromonas gingivalis* and *Prevotella intermedia* [21], as well as cariogenic pathogens such as *Streptococcus mutans* (*S*. *mutans*) [13]. Adding GA (specifically, Acacia Arabica) to toothpaste has been shown to reduce plaque build-up and gingival inflammation [9], this suggested that GA could be used for oral health and maintenance due to its antimicrobial [10, 22, 23], anti-inflammatory [10, 22], biofungicidal, and anticoagulant properties [20].

Oral infections (i.e. dental caries, periodontitis, pulpal, apical, peri-implant diseases, and candidiasis) are a public health problem, with dental caries and periodontitis among the most prevalent diseases globally [6]. The current chemical plaque control strategies have certain limitations, as they may lead to mucosal desquamation, and tooth staining, thus impacting on compliance and efficiency, and causing safety concerns [24]. Hence, natural products are sought as effective alternative antimicrobial agents for plaque control with minimal side effects. The use or incorporation of natural products in these agents is attractive, and could lead to innovative treatment agents in the fight against dental plaque and its consequences [7]. Even more interesting is phytonanotherapy, or the use of nanotechnology to enhance the efficacy and bioavailability of the phytochemicals, which are used as reducing and stabilizing agents in the synthesis of nanoparticles [25]. Nanoparticles (NPs) at a size range between 1 and 100 nm, possess unique physical and chemical properties that found applications in many fields. In medicine, they are used as drug delivery, diagnostic and therapeutic agents [26]. Plant extract-synthesized AgNPs have the potential to prevent and treat dental infections [6]. AgNPs are receiving attention in dentistry due to their antimicrobial activity [6, 27]. Plants are readily available, renewable, safer than the chemical reducing agents in NP synthesis [6, 28, 29], and are potentially less toxic and more environmentally friendly [30, 31]. The broad-spectrum antimicrobial activity of GA-AgNPs [23] encouraged its application in dental therapy. GA-AgNPs have been shown to have activity against pathogenic oral microbes, such as *Escherichia coli* (*E*. *coli*) and *Micrococcus luteus* (*M*. *luteus*) [33], *Staphylococcus aureus* (*S*. *aureus*), *Klebsiella pneumoniae* (K. *pneumoniae*) [34, 35], and *S*. *mutans*[36]. While *S*. *mutans* is fundamental in the induction of dental caries [32], oral infections can be caused by multiple pathogens such as nonstreptococcal bacteria (e.g. *Bifidobacterium* spp., *Scardovia* spp., and *Actinomyces* spp.) and fungi (e.g. *C*. *albicans*) [37]. The aim of the current study was to investigate the antimicrobial effects of GA-AgNPs against 4 different human oral pathogens.

## 2. Materials and Methods

### 2.1. Synthesis and Characterization of Gum Arabic (GA)-AgNPs

#### 2.1.1. Synthesis of GA-AgNPs

GA-AgNPs were synthesized as previously reported [23]. Briefly, 4 mg/mL GAE and two concentrations of AgNO_3_ (0.1 g and 0.4 g) were used to produce GA-AgNPs_0.1g and GA-AgNPs_0.4g, respectively. All reactions were performed in an autoclave at 15 psi at 120°C for 20 min [23].

The GA-AgNPs were centrifuged at 9000 rpm for 45 min and resuspended in sterile deionized water. The AgNPs were stored at room temperature until further characterization. The dry mass was determined by freeze-drying 10 mL of GA-AgNPs on the Virtis Freezer dryer (SP Scientific, Gardiner, NY, USA) and used to calculate their concentrations.

#### 2.1.2. Characterization of GA-AgNPs

The GA-AgNPs were characterized by UV-Vis, DLS, FTIR, and high resolution TEM (HRTEM), as previously described [23, 29]. The GA-AgNPs were diluted 1 : 10 in distilled water and used for analyses.

*(1) UV-Vis Analysis*. The GA-AgNPs were added into a 96 well plate (100 *μ*L), their UV-Vis spectra were measured at 300–650 nm using a POLARstar Omega microplate reader (BMG Labotech, Offenburg, Germany).

*(2) DLS Analysis*. The hydrodynamic diameter, polydispersity index (PDI), and zeta potential of the GA-AgNPs were determined by DLS using a Zetasizer NanoZS90 (Malvern Panalytical Ltd., Malven, UK). The size distribution and PDI of each sample were measured on a cuvette (Malvern Panalytical Ltd), and the zeta potential was measured using a DTS1070 folded capillary cuvette (Malvern Panalytical Ltd). The data were measured in triplicate and represented as the mean particle diameter of the three measurements. The data was analyzed by Zetasizer software version 7.11.

*(3) FTIR Analysis*. FTIR analysis of GA-AgNPs and GA powder were analyzed as previously described [29, 38] using Perkin Elmer Spectrum Two Fourier transform infrared (FTIR) spectrophotometer (Waltham, MA, USA) at the School of Pharmacy (UWC).

*(4) TEM Analysis*. The morphology and core size distribution of GA-AgNPs were examined using TecnaiF20 HR-TEM (FEI Company, Hillsboro, OR, USA) at the Electron Microscope Unit (University of Cape Town, South Africa). One drop of the GA-AgNPs solution was placed onto a carbon coated copper grid and left to dry for a few minutes under a Xenon lamp, as previously described. The core size of the GA-AgNPs was measured from the TEM micrographs by using ImageJ software (http://www.imagej.nih.gov/ij) [39].

### 2.2. Stability Evaluation of the GA-AgNPs

The stability of GA-AgNPs was assessed in water, phosphate buffered saline (PBS), and Müeller–Hinton broth (MHB; Sigma–Aldrich, St Louis, USA) following a previous protocol [40]. Briefly, 200 *μ*L of the GA-AgNPs were mixed with 800 *μ*L of each of the solutions in separate tubes and incubated at 37°C. The stability of the GA-AgNPs was monitored by the UV-Vis spectra of the samples at 1 hour intervals for the first 6 hours, and again at 24, 48, and 72 hours.

### 2.3. Antimicrobial Activity of the GA-AgNPs

The antimicrobial activity of the GA-AgNPs against three bacterial strains: *S*. *sanguinis* (NCTC 7865), *S*. *mutans* (NCTC 10449), *L*. *acidophilus* (ATCC 314), and one fungal strain *C*. *albicans* (ATCC 10231) was determined using the agar disc diffusion and the microdilution assays. The *S*. *sanguinis* and *S*. *mutans* were purchased from Davies Diagnostics (Randburg, Johannesburg, South Africa); and *L*. *acidophilus* and *C*. *albicans* were purchased from the American Type Culture Collection (ATCC; Manassas, Virginia, USA).

All the microbes were cultured on Brain Heart Infusion (BHI) Broth (Sigma–Aldrich), and single colonies were subcultured in BHI agar (Sigma–Aldrich) for all the bacterial strains and Sabouraud dextrose agar for *C*. *albicans* at 37°C for 24 hours. Following the overnight incubation, the microbes were adjusted to the 0.5 McFarland standard (Mcf) using DensiCHEK Plus standards (BioMérieux, Inc., Durham, NC, USA).

#### 2.3.1. Agar Disc Diffusion Method

Sterile 6 mm filter paper discs (Lasec, Cape Town, South Africa) were aseptically infused with 50 *μ*L of each of the treatments: GA-AgNPs at 100 *μ*g/mL, GAE at 4 mg/mL, 0.2% chlorhexidine (CHX), and 5000 units of nystatin. The discs were placed in sterile Petri-dishes and left to air-dry overnight in a laminar flow class 2 cabinets. CHX and nystatin were used as positive controls for bacteria and fungi, respectively; and a sterile disc infused with distilled water was used as a negative control. The microbes at 0.5 Mcf (100 *μ*L of each standardized inoculum) were spread evenly onto the Müeller–Hinton agar (MHA; Sigma–Aldrich), and treatment and control discs were placed on the plate. The plates were incubated for 24 hours at 37°C. Antimicrobial activity was determined by measuring the diameters of the zones of inhibition (ZOI) formed around the paper disc in millimeters using a vernier caliper [23, 41]. The assay was carried out in triplicate for all organisms tested with all treatments on the same plate and repeated three times.

#### 2.3.2. Biofilm Inhibition by Microdilution Method

The microdilution assay was used to determine the minimum inhibitory concentration (MIC), following the M07 guidelines [42] set by the Clinical Laboratory Standards Institute (CLSI). In a 96 well plate, 100 *μ*L of MHB was pipetted into all wells, and 100 *μ*L of the 0.5 Mcf was added in all wells with the exception of the blank well. Following a 24-hour incubation period, the plates were rinsed with PBS three times, and 100 *μ*L of MHB was pipetted into all wells except the blank well. The biofilms were treated with increasing concentrations of GA-AgNPs (1.5625–100 *μ*g/mL), 0.2% CHX, and 5000 units of nystatin. All experiments were conducted in triplicate, and the plates were incubated at 37°C for 24 hours. After treatments, the XTT reduction method was used according to the manufacturer's instructions to measure the biofilm activity, as previously described [43]. The plates were read at 450 nm and 620 nm (reference wavelength) using the SpectroStar Nano microplate reader (BMG Labotech). The MIC_50/90_ were further determined by subculturing 5 *μ*L of each sample on the agar plates and incubated at 37°C for 24 hours following a previous protocol [44]. The total number of colonies appearing on the agar plates was used to determine the MIC_50/90_ for the various treatments.

### 2.4. Adhesion of *S*. *mutans* to Tooth Enamel

Fifty extracted human molar teeth (protocol approved by the Biomedical Research Ethics Committee of the University of the Western Cape, reference number: BM20/1/7) were scaled, cleaned, sonicated, and stored in saline solution at 4°C. The crowns of each extracted tooth were cut into enamel blocks of 5 mm × 5 mm (25 mm^2^) using a diamond disc with irrigation at 10,000 rpm. The enamel blocks received two coats of nail varnish, then were placed inside a 2 mL Eppendorf tube and sterilized in an autoclave for 15 min. The enamel blocks were randomly divided into 5 groups (10 specimens in each group) and incubated with: Group 1: *S*. *mutans* (100 *μ*L Mcf); Group 2: *S*. *mutans* (100 *μ*L Mcf) + GA-AgNPs_0.4g (825 *μ*L); Group 3: GA-AgNPs_0.4g (825 *μ*L); Group 4: *S*. *mutans* (100 *μ*L Mcf) + 0.12% CHX (125 *μ*L); and Group 5: enamel blocks. Then, 1 mL of MHB was added into each tube, and incubated for 24 hours at 37°C. After incubation, the enamel blocks were transferred into tubes containing 1 mL of saline solution.

To determine the surface adhesion of *S*. *mutans* after treatments, the enamel blocks were prepared for scanning electron microscopy (SEM) following a previous protocol [45]. The enamel blocks were fixed in a 0.1% glutaraldehyde solution for 5 min, washed three times with the saline solution and immersed in ethanol (50, 60, 70, 90, 95, and 100%) for 20 min each at room temperature. Aluminium stubs were used to mount the samples. Carbon tabs were placed on the stubs to keep the sample in place. Finally, the enamel blocks were gold coated with a sputtering coater technique (Q 150T ES) for 60 seconds. SEM images were obtained using a field emission SEM (SmartSEM, Zeiss, Germany) operating at 5 kV and 10 μA at the Electron Microscope Unit (University of Cape Town).

### 2.5. Statistical Analysis

The data are presented as the mean ± standard error of the mean of the three independent experiments, which were carried out in triplicate. Statistical analysis was performed by one-way and two-way ANOVA using GraphPad Prism version 6, a value of *p* < 0.05 was considered statistically significant. Finally, post hoc pair-wise testing was carried out to elucidate the statistical differences between two sets of data.

## 3. Results and Discussion

Many regimens for the prevention of dental caries have demonstrated short-lived successes due to their drawbacks, such as mucosal damage and tooth staining [46]. AgNPs have demonstrated antimicrobial activity against several pathogens, including oral microflora, and are now being investigated in the prevention of oral diseases, including dental caries [47]. Their broad spectrum antimicrobial properties, including the fight against drug resistant microbes, has aroused interest in their use in the treatment and prevention of dental caries [46]. In this study, AgNPs synthesized using readily available, affordable, and environmentally friendly GAE were investigated for their antimicrobial activities against oral pathogens.

### 3.1. GA-AgNPs Synthesis and Characterization

GA-AgNPs were synthesized following our optimized protocol as previously reported by Fadaka et al. [23]. The color of the solution was clear upon the addition of GAE into the aqueous solution of AgNO_3_, and changed to dark brown after autoclaving, as shown in Figure 1. The color change was an indication of the formation of GA-AgNPs. This has been reported for GA-AgNPs synthesized using *Acacia Senegal* (L) wild [36], *Gum Acacia* [33], and *Acacia Senegal* [23], the latter being the same species that was used in this study. This confirmed that phytochemicals present in the GAE were able to reduce and stabilize the GA-AgNPs, either individually or collectively [48, 49]. Similar findings were reported for other plant-synthesized AgNPs using plant extracts from *Cotyledon orbiculata* [50], *Salvia Africana Lutea*, *Sutherlandia frutescens* [38], *Justicia glauca* [31], and *Terminalia mantaly* [51], as well as pear fruit extracts [29].

#### 3.1.1. UV-Vis Spectra for GA-AgNPs

UV-Vis spectra confirmed the presence of GA-AgNPs. This method has been one of the most important tools for the characterization of metal nanoparticles (MNPs). It is based on the absorption of light by a sample as a result of the excitation of the surface plasmon vibration in the MNPs [33]. In this study, a UV-Vis spectrum with a surface plasmon resonance (SPR) or maximum absorbance (*λ*_max_) around 400 nm (Figure 2) was indicative of GA-AgNPs formation, which is within the characteristic SPR range for AgNPs [23, 31, 51]. The SPR values were 450 and 425 nm for GA-AgNPs-0.1g and GA-AgNPs-0.4g, respectively. The peak intensity of the GA-AgNPs synthesized with 0.4 g AgNO_3_ was slightly higher than those synthesized with 0.1 g AgNO_3_, which suggested that more AgNPs were formed at this concentration since absorbance is related to the concentration of NPs [51]. The GA-AgNPs_0.1g spectra were broad compared to those of GA-AgNPs_0.4g, which implied that the GA-AgNPs_0.1g were polydispersed [51].

#### 3.1.2. Size Distribution of GA-AgNPs

The hydrodynamic diameter of the GA-AgNPs was 226.4 nm and 220 nm for GA-AgNPs_0.1g and GA-AgNPs_0.4g, respectively (Table 1). The zeta potential of GA-AgNPs_0.1g was −22.9 mV and −24.6 mV for GA-AgNPs_0.4g. Zeta potential is an important parameter that is used to determine the surface charge and the stability of NPs. The zeta potential within the range of +30 mV to −30 mV is considered to be stable, while those outside this range will coalesce due to interparticle van der Waal's attractions. The negative zeta potential of the GA-AgNPs indicated strong repulsion forces between the AgNPs in suspension and will thus prohibit the agglomeration of the AgNPs in solution [52]. The PDI values were 0.060 and 0.156 for GA-AgNPs_0.1g and GA-AgNPs_0.4g, respectively. This confirmed that the AgNPs were uniform and monodispersed, as the PDI values >0.7 suggest that the NPs have a very broad size distribution, while PDI values ≤0.5 are likely to be monodispersed [51].

The HRTEM micrographs in Figure 3 demonstrated that the majority of GA-AgNPs were spherical in shape, with core sizes between 4 and 26 nm. These sizes were smaller than their hydrodynamic sizes, as the latter accounts for both the core size and the molecules that are adsorbed on the surface of the GA-AgNPs, while the HRTEM only represents the core size [51]. Increasing scientific evidence has demonstrated that AgNPs activity depends strongly on their shape and size [53, 54], with the shape being the most relevant physicochemical parameter influencing their bioactivities, including their antimicrobial properties [53]. This was confirmed by the weakest antibacterial activity demonstrated by the silver nanowires when compared with silver nanocubes and nanospheres [54]. In addition, the size of the AgNPs plays an important role in their antimicrobial activity, with smaller sizes showing higher activity than larger AgNPs [54]. This was in line with the current study, where the GA-AgNPs were spherical and had superior antimicrobial activity.

#### 3.1.3. FTIR Analysis of GA-AgNPs

The FTIR spectra of GAE and the GA-AgNPs were compared in order to identify the types of phytochemicals that were involved in the synthesis of the GA-AgNPs.  Figure 4 outlines the similarities between the FTIR spectra of GAE and GA-AgNPs. The GAE showed noticeable peaks at 3514, 2978, 2315, 1628, 1371, and 1065 cm^−1^; the GA-AgNPs_0.4g spectrum showed peaks at 2929, 1615, 1345, and 1077 cm^−1^, while the GA-AgNPs_0.1g showed peaks at 2966, 1638, 1358, and 1041 cm^−1^ (Figure 3). The GAE spectral distribution observed at 3514 cm^−1^ demonstrated the presence of OH stretch; while the 2978 cm^−1^ for GAE, 2929 cm^−1^ for GA-AgNPs_0.4g and 2966 for GA-AgNPs_0.1g indicated the presence of alkanes with C-H bond stretch. The sharp spectral peak at 1628 cm^−1^ for GAE, 1615 cm^−1^ for GA-Ag NPs_0.4g, and 1638 cm^−1^ for GA-AgNPs_0.1g signified the presence of secondary amine NH bend. The spectral peak at the wavelength of 1371 cm^−1^ for GAE, 1345 cm^−1^ for GA-AgNPs_0.4g and 1358 cm^−1^ for GA-AgNPs_0.1g implied organic nitrates. Moreover, another set of peaks representing S = O stretching for sulfoxide in GAE, GA-AgNPs_0.4g, and GA-AgNPs_0.1g were observed at 1065 cm^−1^, 1077 cm^−1^, 1041 cm^−1^, respectively. The variations or shifts in the peak positions of the GAE and GA-AgNPs were observed due to the GAE contribution toward the reduction and stabilization process. The presence of phenols, alcohols, amides, sulfoxide, flavonoids, and steroids was also revealed in other studies using GAE in the synthesis of GA-AgNPs [33, 36].

### 3.2. Stability of GA-AgNPs

The stability of GA-AgNPs was tested in water, PBS, and MHB and measured by their UV-Vis spectral profiles. As shown in Figure 5, the GA-AgNPs were stable in water, PBS, and MHB, as indicated by no changes in the UV-Vis spectra for up to 72 hours. The GA-AgNPs_0.1g was only stable in water and MHB, and revealed signs of instability when subjected to PBS. The GA-AgNPs_0.4g was relatively stable in water, PBS, and MHB.

### 3.3. Antimicrobial Effects of GA-AgNPs on Oral Microbes

In recent years, there has been a growing interest in the use of natural products to fight against drug resistant microbes. This is fueled by the successful use of plant extracts in traditional medicine as a source of antimicrobial agents. GA in particular, has been effective against various periodontal [21] and cariogenic pathogens [13]. In fact, when mixed in water, GA was used as a tooth paste formulation in ancient times, long before commercial toothpastes arrived on the market. Due to its high concentration of calcium and other cations, GA also possesses remineralization effects and prevents caries in enamel lesions [55]. Its use in oral hygiene and health [17] is motivated by its antimicrobial, antioxidant, and anti-inflammatory properties [10, 22], biofilm inhibition and biofungicide activities [20]. These activities are attributed to the presence of flavonoids, chalcones, tannins, phenolic acid, alkaloids, and terpenes in GA [35], and reported to have enhanced activities when used in the bioreduction and synthesis of AgNPs. The NPs penetrate the biofilm structure and release metal ions that destroy the biofilm and inhibit microbial colonization [56].

The antibacterial and antifungal activities of GA-AgNPs and GAE were investigated against three dominant oral pathogens i.e., *S*. *mutans*, *L*. *acidophilus,* and *C*. *albicans*; and one oral commensal species (*S*. *sanguinis*).  Table 2 shows that there were statistical differences in the zones of inhibition (ZOIs) of bacteria exposed to GA-AgNPs_0.1g/0.4g and the positive controls (CHX and nystatin) compared to GAE. There were no ZOIs around the microbes treated with 4 mg/ml GAE and the negative control, indicating that the GAE at the tested concentration had no antimicrobial activity against all microbes tested. This finding was similar to the study conducted by Venkatesham et al. where the GAE from *Gum Acacia* had no antimicrobial activity against *E*. *coli* and *M*. *luteus* [33]. GAE from *Acacia Senegal* showed time and dose-dependent effects against the *S*. *aureus* and *E*. *coli* at 5–40 mg/ml [34]. GAE from *Gum Acacia* and *Acacia Senegal* were also reported to have antibacterial activity against *S*. *aureus*, *E*. *coli*, and *K*. *pneumoniae* at 0.25–2 mg/ml [35] and at 5–40 mg/ml [34], respectively.

The antimicrobial effects of GA-AgNPs_0.1g, GA-AgNPs_0.4g, and CHX were also observed in the nonpathogenic strain (*S*. *sanguinis*), with stronger effects in the *S*. *mutans*, *L*. *acidophilus* and *C*. *albicans*. Generally, the GA-AgNPs_0.4g yielded larger ZOIs compared to GA-AgNPs_0.1g, suggesting that GA-AgNPs_0.4g was more potent. The antimicrobial activity of GA-AgNPs was previously reported against *S*. *mutans,* and the ZOIs at 25, 50, 100, and 200 *μ*g/ml were 14.1 ± 0.7 mm, 15.5 ± 0.8 mm, 16.3 ± 1.0 mm and 18.3 ± 0.5 mm, respectively [36]. In the present study, ZOIs for *S*. *mutans* at 100 *μ*g/ml for GA-AgNPs_0.1g and GA-AgNPs_0.4g were 10.5 ± 0.04 mm and 16.6 ± 0.34 mm, respectively. Studies have reported that the bactericidal properties of AgNPs are size and shape-dependent [57], where the smaller size AgNPs presents a larger surface area which is ideal for interaction with the bacterial cell wall [58].

The MIC_50_ and MIC_90_ for the two GA-AgNPs were determined from the microdilution assay, and by subculturing a sample from each well. MIC_50_ and MIC_90_ were defined as the lowest concentration, which inhibited 50% and 90% of the growth when compared with the untreated microbes, respectively [59]. The MIC_50_ and MIC_90_ for GA-AgNPs_0.4g against all microbes (*S*. *sanguinis*, *S*. *mutans*, *L*. *acidophilus*, and *C*. *albicans*) were 8-fold lower than that of GA-AgNPs_0.1g; at 3.125 and 12.5 *μ*g/ml, respectively (Table 3). The GA-AgNPs_0.4g had higher ZOIs and lower MICs than GA-AgNPs_0.1g across the tested microbes. This indicated that GA-AgNPs_0.4g were more effective than the GA-AgNPs_0.1g. This effect can be correlated with their small size, as illustrated in Figure 3. The smaller AgNPs had higher antimicrobial activity than the larger particles as corroborated by Lu et al. [54]. In our previous study, we demonstrated the broad spectrum antibacterial activity of GA-AgNPs_0.4g with a MIC of 6.25–25 *μ*g/ml against a number of human pathogens, namely, *S*. *aureus*, MRSA, *S*. *epidermidis*, *S*. *pyogenes*, *K*. *pneumoniae,* and *E*. *coli* [23]. Independent studies also reported the potency of GA-AgNPs against an oral pathogen (*S*. *mutans*) with MIC of 10.0 *μ*g/mL [36], and between 1.625 and 3.25 *μ*g/mL against the fish bacterial pathogens (*Aeromonas hydrophila* and *Pseudomonas aeruginosa*) [60].

### 3.4. GA-AgNPs Prevents *S*. *mutans* Adhesion Biofilm Formation on Tooth Enamel

For dental application, AgNPs must have the ability to attach themselves to the enamel surfaces for extended activity. In this work, we evaluated the adherence capacity of *S*. *mutans* on the healthy human dental enamel when it was first exposed to the GA-AgNPs_0.4g. The surface of the enamel was colonized by the *S*. *mutans* biofilm when no treatment was added (Figure 6(a)). The SEM micrographs indicated that the application of GA-AgNPs_0.4g made the enamel appear smoother, and prevent bacterial colonization (Figure 6(b)). There was no bacterial growth in Figures 6(b)–6(d), the texture of the enamel exposed to GA-AGNPs (Figures 6(b) and 6(c)) appeared to be smoother compared to the CHX-treated enamel (Figure 6(d)) and the vehicle enamel (Figure 6(e)). These results imply that the GA-AgNPs_0.4g may have the ability to prevent attachment of *S*. *mutans* on the teeth. Similarly, adding AgNPs to the commercial adhesive systems changed the texture of the enamel [61], which might also prevent colonization of the enamel by bacteria. In other studies, *S*. *mutans* biofilm treated with chemically synthesized AgNPs presented apparent structural destruction, suggesting that biofilm formation was inhibited [45]. The GA-AgNPs presented similar effects to that of CHX, and prevented the attachment of *S*. *mutans* biofilm, which suggested that AgNPs can be added to dental care products to prevent infections.

## 4. Conclusions

The plant extract-mediated synthesis of AgNPs has emerged as a new avenue to produce biocompatible AgNPs. The findings in this study suggest that GA-AgNPs are promising antimicrobial agents against oral microbes. The GA-AgNPs_0.4g had enhanced antimicrobial activity compared to GA-AgNPs_0.1g. Therefore, the GA-AgNPs can be used as an additive to dental products, particularly because it can attach itself to enamel and prevent bacterial biofilm formation on the teeth.

## Figures and Tables

**Figure 1:** Synthesis of GA-AgNPs using an autoclave method. The solutions containing AgNO_3_ and GAE for the synthesis of GA-AgNPs_0.1g and GA-AgNPs_0.4g, before and after autoclaving for 20 min.

**Figure 2:** UV-vis analysis for GA-AgNPs.

**Figure 3:** (a) HRTEM micrographs and (b) core size distribution of the GA-AgNPs.

**Figure 4:** FTIR images of GAE, GA-AgNPs_0.4g, and GA-AgNPs_0.1g.

**Figure 5:** UV-vis spectra of (a) GA-AgNPs_0.1g; and (b) GA-AgNPs_0.4g in water, PBS, and MHB measured over a 72 hour period.

**Figure 6:** Exposure of GA-AgNPs_0.4g to *S*. *mutans* inhibits bacterial adhesion on the enamel surfaces. (a) Tooth enamel with *S*. *mutans* without treatment, (b) with GA-AgNPs_0.4g with *S*. *mutans*, (c) GA-AgNPs_0.4g without bacteria, (d) *S*. *mutans* and CHX D), (e) tooth enamel without bacteria and treatment.

**Table 1:** DLS analysis of GA-AgNPs.

Samples	Hydrodynamic size (nm)	PDI	Zeta potential (mV)
GA‐AgNPs_0.1g	226.4	0.060	−22.9
GA‐AgNPs_0.4g	220	0.156	−24.6

**Table 2:** ZOIs as a measure of antimicrobial activity of GA-AgNPs.

Microbes	ZOIs (mm)				
	GAE	GA-AgNPs_0.1g	GA-AgNPs_0.4g	0.2% CHX	Nystatin
*S*. *sanguinis*	0	9.96 ± 0.09	13.38 ± 0.10	19.74 ± 0.08	
*S*. *mutans*	0	10.48 ± 0.04	16.62 ± 0.34	22.65 ± 0.05	
*L*. *acidophilus*	0	9.77 ± 0.02	13.92 ± 0.20	18.53 ± 0.10	
*C*. *albicans*	0	12.44 ± 0.28	17.97 ± 0.41		22.86 ± 0.01

**Table 3:** MICs values for the GA-AgNPs.

Microbes	MIC_50_ (*μ*g/ml)		MIC_90_ (*μ*g/ml)	
	GA-AgNPs_0.1g	GA-AgNPs_0.4g	GA-AgNPs_0.1g	GA-AgNPs_0.4g
*S*. *sanguinis*	25	3.125	100	12.5
*S*. *mutans*	25	3.125	100	12.5
*L*. *acidophilus*	50	3.125	100	12.5
*C*. *albicans*	50	3.125	100	12.5

## Data Availability

The data are presented as tables and figures in the manuscript.
